# Community’s perceived high risk of coronavirus infections during early phase of epidemics are significantly influenced by socio-demographic background, in Gondar City, Northwest Ethiopia: A cross-sectional -study

This article has been retracted.

**DOI:** 10.1371/journal.pone.0242654

**Published:** 2020-11-19

**Authors:** Gebisa Guyasa Kabito, Mekuriaw Alemayehu, Tesfaye Hambisa Mekonnen, Sintayehu Daba Wami, Jember Azanaw, Tsegaye Adane, Zelalem Nigussie Azene, Mehari Woldemariam Merid, Atalay Goshu Muluneh, Demiss Mulatu Geberu, Getahun Molla Kassa, Melaku Kindie Yenit, Sewbesew Yitayih Tilahun, Kassahun Alemu Gelaye, Habtamu Sewunet Mekonnen, Abere Woretaw Azagew, Chalachew Adugna Wubneh, Getaneh Mulualem Belay, Nega Tezera Assimamaw, Chilot Desta Agegnehu, Telake Azale, Animut Tagele Tamiru, Bayew Kelkay Rade, Eden Bishaw Taye, Asefa Adimasu Taddese, Zewudu Andualem, Henok Dagne, Kiros Terefe Gashaye

**Affiliations:** 1 Department of Environmental and Occupational Health and Safety, Institute of Public Health, College of Medicine and Health Sciences, University of Gondar, Gondar, Ethiopia; 2 Department of Women’s and Family Health, School of Midwifery, College of Medicine and Health Sciences, University of Gondar, Gondar, Ethiopia; 3 Department of Epidemiology and Biostatistics, Institute of Public Health, College of Medicine and Health Sciences, University of Gondar, Gondar, Ethiopia; 4 Department of Health Systems and Policy, Institute of Public Health, College of Medicine and Health Sciences, University of Gondar, Gondar, Ethiopia; 5 Department of Psychiatry, College of Medicine and Health Sciences, University of Gondar, Gondar, Ethiopia; 6 Department of Medical Nursing, School of Nursing, College of Medicine and Health Sciences, University of Gondar, Gondar, Ethiopia; 7 Department of Pediatric and Child Health Nursing, School of Nursing, College of Medicine and Health sciences, University of Gondar, Gondar, Ethiopia; 8 School of Nursing, College of Medicine and Health Sciences and Comprehensive Specialized Hospital, University of Gondar, Gondar, Ethiopia; 9 Department of Health Education and Behavioral Sciences, Institute of Public Health, College of Medicine and Health Sciences, University of Gondar, Gondar, Ethiopia; 10 Department of General Midwifery, School of Midwifery, College of Medicine and Health Sciences, University of Gondar, Gondar, Ethiopia; 11 Department of Clinical Midwifery, School of Midwifery, College of Medicine and Health Sciences, University of Gondar, Gondar, Ethiopia; 12 Department of Gynecology and Obstetrics, University of Gondar College of Medicine and Health Sciences, Gondar, Ethiopia; Jamia Hamdard, INDIA

## Abstract

**Background:**

Epidemiological studies during the early phase of the coronavirus (COVID-19) pandemics reported different level of people’s risk perception in different countries. There is a paucity of data on perceived high risk of COVID-19 and associated factors in Ethiopia. We sought to assess the prevalence of community’s perceived high risk about COVID-19 infections and associated factors among Gondar town community.

**Methods:**

A cross-sectional study was carried out from April 20 to 27, 2020 in Gondar town community, Northwest Ethiopia. Multistage cluster sampling technique was used to recruit 635 participants. Structured and pre-tested questionnaire was used to collect the data. Descriptive statistics, bivariate and multivariable binary logistic regression were used to summarize the results.

**Results:**

A total of 623 participants were considered in the analysis with a response rate of 98.1%. The prevalence of coronavirus high risk perceptions of the respondents was found to be 23.11% (95% CI; 19.80%–26.43%). Age above 45 years (AOR = 1.41, 95%CI; 1.19–2.66), college and above educational level (AOR = 0.28, 95%CI; 0.21–0.98), and poor knowledge towards COVID-19 virus (AOR = 1.57, 95%CI; 1.09–2.23) were significantly associated with perceived high risk about COVID-19.

**Conclusions:**

The prevalence of perceived high risk of COVID-19 was found to be low. Factors such as age, educational status, and knowledge about COVID-19 virus were found to be independent predictors of perceived high risk towards COVID-19. Government and non-government organizations should use formal and informal means of educating the community.

## Introduction

The novel coronavirus disease (COVID-19) and its causative virus, severe acute respiratory syndrome coronavirus (SARS-CoV-2), have identified the world since December 2019 [1]. WHO declared the outbreak of COVID-19 a pandemic on 11 March 2020 [2], with millions of people infected and hundreds of thousands deaths [3]. At the time of this writing (July 27, 2020), there are 13,968 cases of COVID-19 in the Ethiopia with 223 deaths [4]. COVID-19 therefore affects mainly a common good which is public health [5]. On top of this, many adverse consequences exist in an environment that interconnected from local to international scales outside the health systems, including production interruptions; intense economic consequences [6, 7], and everything about human life, including exports and imports of goods, business, infrastructural development, agriculture, and education look stopped [8].

While the number of deaths from the disease is growing around the world, understanding people’s risk perception is becoming increasingly relevant to better inform messaging and policies [9]. As the people’s understanding of risk of a pandemic leads to increased public engagement in preventive action [10]. Risk perceptions described as an implicit assessments of the hazards to which people are or might be exposed [11], including a multitude of detrimental effects that people associate with a particular cause [12]. A broad spectrum of studies over recent decades has shown that risk perception is a subjective psychological system shaped by cognitive, emotional, social, cultural and individual differences both between individuals and countries [13].

A few epidemiological studies during the early phase of the COVID-19 epidemics reported the levels of people’s risk perceptions were different from low in America [3] to very high in South Africa [14]; a high risk perception in Hong Kong [15] to Malaysia was reported [16], and in Ghana 68.3% perceived risk of COVID-19 infection [17]. Moreover, there are aspects of pandemics that can increase the perception of risk, so-called dread factors that are largely relevant to the current SARS-CoV-2 pandemic [18, 19]. These include high infection levels, severe morbidity and mortality, lack of protective or therapeutic interventions, and rapid rises in cases or case-fatality rates [18, 20]. On the contrary, the lack of understanding around COVID-19 has shaped public perception and response, with some in the public becoming extremely anxious, although others restrained risks by equating it to something more familiar such as influenza [21].

In developing countries including Ethiopia there is a paucity data of risk perceptions for the current COVID-19 epidemics; assumed COVID-19’s ongoing rampant nature. Therefore, this study aimed to analyze the prevalence and factors associated with risk perception of COVID-19 infections among residents in Gondar town, Northwest Ethiopia.

## Materials and methods

### Study design, period, and area

A community-based cross-sectional study design was applied to evaluate level of risk perception regarding COVID-19 and predictors among a sample of residents in Gondar city from April 20 to 27, 2020. The city is located in the state of Amhara, 750 km far from the North West of Addis Ababa, the capital city of Ethiopia. Gondar had 22 Kebeles, with an estimated 360,600 population [22]. At the time of this study, 51,304 households were registered.

### Source and study populations

All people who reside in Gondar city were the source population. The randomly selected residents in the selected Kebeles were our study population. Residents living in selected households as heads or any other household members ≥18 years of age were included in the study and those who were unable to communicate easily during data collection were excluded.

### Sample size determination and sampling procedures

The single population proportion formula [23] was used to determine the sample size with the following statistical assumptions: *p* (proportion of risk perception assumed to be 50% since this would yield the maximum sample size),), *d* (margin of error = 5%) and *Zα/2* (standard score value for 95% confidence level = 1.96). By considering 10% non-response rate and design effect of 1.5 the final sample size was 635. We used multistage household cluster sampling technique to recruit eligible samples. Eight Kebeles were selected out of 22 Kebeles randomly. Namely Kebele 7, Kebele 8, Kebele 9, Kebele 13, Kebele 16, Kebele 17, Kebele 18, Kebele 20 were selected by using lottery method, then from each Kebele one to two Ketena/s (the lowest administrative cluster) were selected depending on the number of households. The selected Ketena/s were considered as cluster and all households in the selected Ketena were included. Either parents in the household was interviewed or one family member age above 18 year was the respondent in the household whenever the parents are not available at the time of data collection. Data collection was carried out by following all the precautionary mechanisms that recommended by WHO i.e. Physical distancing, face mask, and hand hygiene.

### Data collection tools and variable measurement

Data were collected using a pre-tested and structured interviewer-administered data collection methods. We adopted and modified survey questionnaires from previous studies on similar subject about COVID-19 [15–17, 24]. The outcome variable of this study, risk perception towards COVID-19 infection was measured by two psychological dimensions; perceived susceptibility and perceived severity. The first dimension was proxied by how likely one considered oneself (his/her families) would be infected with COVID-19 if no preventive measure will be taken. The second dimension was proxied by how one rated the seriousness of symptoms caused by COVID-19, their perceived chance of having COVID-19 cured and that of survival if infected with COVID-19. By combining the two dimension, five items with five responses options were asked to determine the respondents’ levels of risk perception. Responses were scored on a five-point ordinal scale reflecting the levels of contacting COVID-19, such as "How likely you will be infected? How likely your family will be infected?" Every item on a scale from 1 to 5, ranges in the susceptibility from ‘very unlikely’ to ‘very likely'. To assess the perceived severity the participant was asked ‘the seriousness of symptoms caused by SARS-CoV-19, chance of having COVID-19 cured, chance of survival if infected with COVID-19’ on a five-point ordinal scale reflecting the severity of COVID-19, from ‘not serious at all’ to ‘very serious’ and ‘Very low’ to ‘very high’. Responses were dichotomized into low perceived risk (“very unlikely” or “unlikely”), (“very low” or “low”), and (“not serious at all” or “not serious”) and high perceived risk (“very likely” or “likely”) [25]. The Cronbach’s alpha coefficients of the perception items were 0.74 and demonstrated that the internal consistency of perception items was satisfactory [26].

To measure knowledge about COVID-19, 13 items were adapted from previous research [27]. These items include the participant knowledge about clinical presentations (items 1–4), transmission routes (items 5–8) and prevention and control (items 9–13) of COVID-19. Participants were given “true,” “false,” or “not sure” response options to these items. A correct response to an item was assigned 1 point, while an incorrect/not sure response was assigned 0 points. Participants who responds median and above score of the knowledge questions about COVID-19 were labeled as having good knowledge otherwise poor knowledge.

To assess attitudes about COVID-19, 8 items were asked on a five-point ordinal scale “strongly disagree” to “strongly agree”. Participants who responds median and above score of the attitude questions about the COVID-19 were labeled as having favorable attitude otherwise unfavorable attitude. Moreover, several demographics were included: age, gender, marital status, occupational status, monthly income, family size, education level and religion. They were also asked about their self-perceived health condition, participants were asked, ‘How would you describe your current health condition?’, and the participants chose a score from 1 to 5, ranging from ‘My health condition is very bad’ to ‘My health condition is very good’. Presence of respiratory symptoms in the past 14 days was also asked with Yes/No response. The full survey questionnaire is provided in the S1 Appendix.

### Data quality control

The instrument was initially prepared in English and then translated into the local language, Amharic and back translated to English in order to check its consistency. The questionnaires were administrated in Amharic. We recruited twenty four data collectors and six supervisors with different health-related professional backgrounds. Two days training was offered for data collectors and supervisors on topics related to research objectives, clarity of questions, utilization of PPE, the confidentiality of information and consent in the study. The training was given in lecture, roleplay and discussion ways. The questionnaires were pre-tested on 30 samples that were not included in the final analysis and the relevant modifications were made before the actual data collection was conducted.

### Data management and statistical analysis

The data were checked for completeness and entered into Epidata version 4.6, and exported to STATA 14 windows for analysis. Frequency distributions, percentages, means, and standard deviations were used for description of the results. Binary logistic regression (Bivariable and multivariable binary logistic regression) was performed to identify statistically significant variables using a cut-off p< 0.2 in the bivariable analysis to identify candidate variables for multivariable logistic regression. Adjusted odds ratio with 95% confidence interval was used to declare statistically significant variables on the basis of p<0.05 in the multivariable binary logistic regression model. Hosmer and Lemeshow goodness-of-fit test was used to check the model fitness (P>0.05).

### Ethics approval and consent to participate

Ethical clearance was obtained from the Institutional Review Board (IRB) of University of Gondar and an official permission letter was gained from the city administrative office. Written informed consent was obtained from each participant before conducting the actual data collection process. Any identifiable issues were eliminated to ascertain confidentiality. Further more appropriate infection prevention practices and principles related with COVID-19 were considered during data collection process. Data collectors provided health education for the household after the interview has been completed based on the gaps identified as appropriate.

## Results

### Socio-demographic characteristics of the participants

Out of 635 selected samples, 623 of whom completed the interviews with a response rate of 98.1%. A high proportion of the respondents were female (402, 64.53%). The mean age (±SD) was 36.3 (±13.2) years, ranging from 18 to 80 years. Among them, (202, 32.42%) have received college-level education or above, (195, 31.30%) have complete secondary school education, (101, 16.21%) have finished primary school and (125, 20.06%) did not receive any formal education. Around two-third of the study participants were married (373, 59.87%). Regarding occupation, nearly three-fourth (448, 71.91%) of the participants were unemployed. More than half of the participants (320, 51.36%) had a monthly income of less than 2500 Ethiopian Birr (ETB, 35 Ethiopian Birr = 1$USD) and (303, 48.64%) reported their monthly income was greater or equals to 2500 ETB. On average, 4 and above people lived in the same household at the time of the study (SD = 2.04, min = 1, max = 14) (Table 1).

**Table 1:** Socio-demographic characteristics of respondents among residents in Gondar city, Northwest Ethiopia, 2020.

Variables(n = 623)	Frequency (n)	Percent (%)
**Sex**		
Male	221	35.47
Female	402	64.53
**Age in years**		
18–26	163	26.16
27–33	150	24.08
34–45	174	27.93
Above 45	136	21.83
**Educational status**		
No formal education	125	20.06
Primary school	101	16.21
Secondary school	195	31.30
College and above	202	32.42
**Marital status**		
Unmarried	250	40.13
Married	373	59.87
**Average household income (ETB)**		
<2500	320	51.36
> = 2500	303	48.64
**Occupational status**		
Unemployed	448	71.91
Employed	175	28.09
**Family number in HH**		
Less than 4	316	50.72
4 and above	307	49.28
**Religion**		
Orthodox	433	69.50
Muslim	154	24.72
Protestant	27	4.33
Others^a^	9	1.44

Keys:

^a^ = Catholic, Jewish;

ETB = Ethiopian Birr (currency);

HH = Households.

### Respondents’ levels of knowledge, attitudes towards coronavirus and self-perceived health conditions

In this study half (50.7%) of participants had good knowledge about COVID-19. About 57.5% and 52% of participants had favorable attitude towards COVID-19 and its preventive measures respectively. Majority (52.33%) of participants were had very good perceived health status (Table 2).

**Table 2:** Levels of knowledge, attitudes towards coronavirus and self-perceived health conditions of respondents among residents in Gondar city, Northwest Ethiopia, 2020.

Variables (n = 623)	Frequency (n)	Percent (%)
**Self-perceived health conditions**		
Very good	326	52.33
Good	238	38.20
Fair	43	6.90
Bad	13	2.09
Very bad	3	0.48
**Medical consultation within two weeks**		
Yes	66	10.59
No	557	89.41
**Respiratory symptoms within two weeks**		
Yes	74	11.88
No	549	88.12
**Knowledge towards COVID-19 virus**		
Poor	307	49.28
Good	316	50.72
**Attitude towards COVID-19 virus**		
Unfavorable	265	42.54
Favorable	358	57.46

### Prevalence of perceived risk of coronavirus (COVID-19)

The overall prevalence of coronavirus high risk perceptions of the respondents was found to be 23.11% (N = 144), 95% CI (19.80%–26.43%).

### Factors associated with perceived risk of COVID-19

In a bivariate binary logistic regression analysis, factors including sex, educational status, age, family size, occupational status, average household income, knowledge and attitudes towards COVID-19 virus were explored to significantly influence the levels of risk perceptions towards COVID-19. After controlling for confounders in a multivariable logistic regression analysis, age, educational status, and knowledge about COVID-19 remained to significantly influence the perception of risk towards COVID-19 (Table 3).

**Table 3:** Factors associated with perceived risk of coronavirus among residents in Gondar city, Northwest Ethiopia, 2020.

Variable (N = 623)	Risk perception of COVID-19 infection		COR(95%CI)	AOR (95%CI)
	low	high		
**Sex**				
Male	178	43	1	1
Female	301	101	1.39 (0.93, 2.08)	1.20 (0.78, 1.83)
**Age**				
18–26	130	33	1	1
27–33	117	33	1.11 (0.65, 1.91)	1.10 (0.63, 2.11)
34–45	142	32	0.89 (0.52, 1.53)	0.77 (0.43, 1.38)
Above 45	90	46	2.01 (1.20, 3.39)	1.41 (1.19, 2.66) **
**Educational level**				
No formal education	80	45	1	
Primary education	73	28	0.68 (0.39, 1.20)	0.62 (0.37, 1.59)
Secondary education	153	42	0.49 (0.30, 0.80)	0.44 (0.29, 1.19)
College and Above	173	29	0.30 (0.17, 0.51)	0.28 (0.21, 0.98) **
**Average household income (ETB)**				
<2500	230	90	1.80 (1.23,2.64)	1.38 (0.90, 2.09)
> = 2500	249	54	1	
**Occupation status**				
Employed	146	29	1	
Unemployed	333	115	1.74 (1.11, 2.73)	1.14 (0.67, 1.94)
**Knowledge towards COVID-19 virus**				
Poor	223	84	1.61 (1.10, 2.34)	1.57 (1.09, 2.23) ***
Good	256	60	1	
**Attitude towards COVID-19 virus**				
Unfavorable	200	65	1.15 (0.79, 1.67)	0.97(0.65, 1.45)
Favorable	279	79	1	

Keys:

**statistically significant at p < 0.01|

***statistically significant at p < 0.0001|

Hosmer and Lemeshow test = 0.854 showed that the model fitted well.

## Discussion

This study aimed on determining the prevalence of community’s perceived risk of coronavirus infections during early phase of epidemics and associated factors. As a result, the prevalence of coronavirus high risk perception was 23.11%and factors such as age, educational status, and knowledge about COVID-19. This is in line with other studies which showed socio-demographic factors might have an effect on perceived risk coronavirus infection [17, 28, 29].

This study is almost similar with the previous findings reported in the UK (26.4%) [30] and Austria (19%) [31]. However, the result of our finding was higher than the study done in India (7.6%) [32]. Moreover, in contrast to our findings, a number of studies reported remarkably higher levels of risk perception towards COVID-19, such as in Iraq (43.6%) [33], Thailand (75%) [24], China (91%) [34], and Ghana (67.4%) [17]. Such similarities and variations possibly might be due to differences in study design, data collection tools and procedures, study period, measurements of the variables (categorization into binary, tertiary and quartile). As well, differences in socio-demographic backgrounds, levels of mass media utilization, individual differences, economic and cultural difference, and levels of risk communication of the governments could affect either positively or negatively the level of risk perceptions towards COVID-19. Furthermore, this might be due to the creeping nature of this kind of hazard, which begins to concern only when the negative effects of the trigger factor become visible and tangible and the emergency could already have reached the critical transition, shifting in a cascading disaster [5]. In addition to this, particularly, previous studies suggest that the spread of a virus can contribute to a widespread sense of risk in the community [35].

Age of the study participants was found to be significantly associated with perceived high risk for COVID-19. Study participants with age above 45 years had 1.41 times (95%CI; 1.19–2.66) risk of experiencing high perceived risk towards COVID-19 than participants ageless than 26 years old. This finding was in-line with a finding reported by a review [36], being older is associated with a higher chance of adopting preventive behavior during pandemic due to greater level of susceptibility and perceived severity of disease. This study also gives additional evidence on high perceived risk towards COVID-19 pandemic and this evidence helps to identify the target group for the intervention.

Educational status of the study participants was found to be significantly associated with perceived high risk for COVID-19. Participants with college and above educational status had 72% lower perceived high risk for COVID-19 compared with participants with no formal education. The possible explanation for this might be due to the participants with high education background has a better understanding to apply the precaution measures to prevent the risk of the pandemic so that they had lower perceived risk for the pandemic. This is in line with the findings of several studies [37–39] reported that those with more education are more likely to adopt precautionary behaviors to protect themselves against different pandemics.

Knowledge towards COVID-19 virus was found to be associated with perceived high risk for COVID-19. Participants who have poor knowledge towards COVID-19 virus had 1.57 times risk for perceived high risk for COVID-19 compared with those participants who have a good knowledge. In contrast to this finding, college students in China [29] with higher knowledge level have higher risk perceptions (P<0.01). This is not meant strict comparison, however, participants in this study at community level of minimal information sources compared to college students and there may also be additional differences of perception COVID-19 beliefs. Nevertheless, the higher knowledge of COVID-19, the more knowledge about its transmission, sign and symptoms, preventive measures, the more they can fully understand the power of COVID-19 infection, improve risk of perception, and the disease is hidden and difficult to identify [40, 41], the risk perception level is higher.

These study findings should be interpreted with the following limitations. The questionnaire was administered through face-to-face interview and it might have resulted socially acceptable responses. Therefore, social desirability bias might have been introduced.

## Conclusions

The prevalence of perceived high risk of COVID-19 was found to be low. Factors such as age, educational status, and knowledge about COVID-19 virus were found to be independent predictors of perceived high risk towards COVID-19. To increase perceived high risk of coronavirus, the government and non-government organizations should use both formal and non-formal means of educating the community.

## Supporting information

S1 Appendix Full survey questionnaire. (DOCX)

S1 Dataset This is data set used in analysis. (XLS)

## Abbreviations

AOR: Adjusted Odds Ratio
CI: Confidence Interval
COR: Crude Odds Ratio
COVID-19: Corona virus disease 19
ETB: Ethiopia Birr
OR: Odds Ratio
SD: Standard Deviation
STATA: Statistics and Data
WHO: World Health Organization
